# Neural Network-Based Beam Pumper Model Optimization

**DOI:** 10.1155/2022/8562387

**Published:** 2022-05-09

**Authors:** Dehua Feng, Yaoguang Qi, Yanqun Yu, Hongying Zhu

**Affiliations:** College of Mechanical and Electronic Engineering, China University of Petroleum (East China), Qingdao 266580, China

## Abstract

Beam pumper is the earliest and most popular rod pumper driven by surface dynamic transmission devices. Drawing on modern theories and methods of industrial model design, the model optimization of beam pumper could promote the diversity, serialization, standardization, generalization, precision balance, and energy reduction of beam pumper design. Therefore, this study tries to optimize the model of beam pumper based on a neural network. Specifically, the system efficiency of beam pumper was decomposed, the surface and downhole working efficiencies were analyzed, and the model optimization flow was explained for beam pumper. Then, a radial basis function (RBF) neural network was established and trained by the sample data on beam pumper model. Besides, the mapping between model parameters and the optimization objective (system efficiency) was constructed. Moreover, the authors summed up the model optimization contents of beam pumper and predicted the relevant parameters of model optimization. The results demonstrate the effectiveness of our model.

## 1. Introduction

Beam pumper is the earliest and most popular rod pumper driven by surface dynamic transmission devices [1–4]. It has long attracted the attention of sci-tech researchers. In the past two decades, more and more new beam pumpers have been developed and put into production [5–11]. A key link of the research and development (R&D) for new beam pumpers is to fully consider the structural performance indices of the pumper, strike a balance between pumper model, pumper functions, and production efficiency, and maximize the economic value of the beam pumper [12–16]. Beam pumper designers are faced with a major task: optimize the model of beam pumper by modern theories and methods of industrial model design, without changing the working performance of beam pumper [17–21]. The model optimization could promote the diversity, serialization, standardization, generalization, precision balance, and energy reduction of beam pumper design.

Considering the rods, tubes, and liquid columns of beam pumper, Zi-Ming et al. [22] established a three-dimensional (3D) dynamic model, which can be expressed as a set of partial differential equations. To make the model more reasonable, an experiment was carried out on South 1-2-22 Well in Daqing Oilfield, and the calculated torque curve was contrasted with the measured torque curve. The experimental results show that the 3D dynamic model is highly accurate and precise and applicable to the design and optimization of the structure and well operation of the beam pumper. Gu et al. [23] modeled and optimized beam pumper by an artificial neural network (ANN). The optimization was realized with Strength Pareto Evolutionary Algorithm 2 (SPEA2). In this way, the optimal set of operation parameters was obtained, which maximizes the oil production, and minimizes power consumption. Li et al. [24] proposed a new particle swarm optimization (PSO) algorithm based on chaotic search and introduced it into the optimal design of beam pumper. The new PSO takes the minimum peak torque factor of the stroke of the beam pumper as the objective function, providing a novel way for the design of complex structures. Based on the API-RP-11L design guidelines, Yang et al. [25] put forward a design optimization method for beam pumper. Their method not only offers an efficient and rapid optimization tool for the modular design of beam pumper but also provides an overall design formula that meets the API design specifications. Drawing on the domestic research of the modular design of beam pumper, Niu [26] suggested combining beam pumper modularization with parametric design. Following the function method, the main structural parameters were collected from the serial module division and subjected to parametric design. The overall performance of the design results was tested and analyzed from both kinematics and kinetics.

The current research of industrial model design and optimization mostly targets cars, home appliances, and computer numerically controlled (CNC) machine tools. The studies on beam pumper mainly focus on shape optimization issues like kansei engineering, and the introduction of emotional factors. There is no report that predicts and optimizes the model parameters of beam pumper based on the results of system efficiency analysis. Therefore, this study attempts to optimize the model of beam pumper based on a neural network. The main contents are as follows: (1) The system efficiency of beam pumper was decomposed, and the surface and downhole working efficiencies were analyzed. (2) The model optimization flow was explained for a beam pumper. (3) A radial basis function (RBF) neural network was established and trained by the sample data on beam pumper model. Besides, the mapping between model parameters and the optimization objective (system efficiency) was constructed. (4) After summing up the contents of beam pumper model optimization, the authors predicted the relevant optimization parameters, selected the best optimization scheme, and evaluated the effect of the scheme through field test. The proposed model was proved effectively through experiments.

## 2. System Efficiency Analysis

The model structure of beam pumper is illustrated in Figure 1, where 1–12 represent skid base, motor, crank counterweight, connecting rod, crank, reduction box, latching beam, rear support, beam, horsehead, beam hanger, and bracket, respectively.

The system efficiency of beam pumper is defined as the ratio of the energy consumed by the pumper to lift the oil to the total energy consumption of the pumper. Based on the system efficiency analysis, the model parameter optimization of beam pumper can be viewed as a multiobjective optimization problem. The traditional approximation model and optimization algorithm can effectively optimize the model parameters of some beam pumpers, but the optimization effect is dampened by their undesirable prediction accuracy. To predict and optimize the model parameters of beam pumper from the perspective of energy conservation, the first step is to decompose the system efficiency of beam pumper and analyze the energy-saving mechanism.

Through stepwise analysis on efficiency decomposition of beam pumper, this study obtains the indices affecting the efficiency, finds the way to enhance the efficiency, and identifies the main indices for energy conservation of beam pumper. The balance and energy consumption of beam pumper were systematically analyzed, laying a solid theoretical basis for further improvement of beam pumper. The efficiency analyses are as follows:

The system efficiency *δ*_*a*_ of beam pumper is the product between the surface working efficiency *δ*_*b*_ and the downhole working efficiency *δ*_*c*_:

(1) $$\begin{array}{c} \delta_{a}=\delta_{b}\times \delta_{c}. \end{array}$$

The surface working efficiency of the pumper is the integrated efficiency of pumper components such reduction box, motor, and rod under normal conditions. The downhole working efficiency refers to the integrated efficiency of the core downhole components, such as sucker rod, tubing string, sealing device, and deep well pump.

Among them, the motor efficiency is the input–output power ratio of the motor. It includes several forms of energy loss, such as copper loss, iron loss, and heat dissipation. The copper loss is equal to the product of the square of the current and the resistance. The iron loss is the loss of energy due to the resistance of ferrous materials during the change of magnetic field poles. The output efficiency of the belt of the reduction box is usually defined as the ratio of the output power of the reduction box to that of the motor, which is normally greater than 85%. The efficiency of the belt consists of wear power and deformation power. Let *R*_*y*_ be the longitudinal curved elastic modulus of the belt; *J* be the cross-sectional inertial moment of the belt; *m* be the rotation speed of the belt; *β* be the wrap angle of the belt. Then, the wear power can be calculated by

(2) $$\begin{array}{c} \Delta T_{1}=\frac{R_{y}}{J}\times \frac{\pi m}{30\beta }\times 10^{-3}. \end{array}$$

Let Δ*T*_2_ be the power loss induced by belt deformation; *u* be the linear speed of the belt; *X* be the cross-sectional area of the belt; *R*_*K*_ be the tensile elastic modulus of the belt; and *G* be the tension of the belt. Then, the deformation power can be calculated by

(3) $$\begin{array}{c} \Delta T_{2}=\frac{G^{2}u}{R_{K}X}\times 10^{-3}. \end{array}$$

The efficiency of reduction box is composed of its bearing operation efficiency, and box member loss. Let *H*, *u*_*e*_, and *g* be the load, linear speed, and friction coefficient of the bearing, respectively. Then, the frictional power loss *T*_*c*_ of the supplementary bearing can be calculated by

(4) $$\begin{array}{c} T_{c}=96Hu_{e}g. \end{array}$$

Let *g* be the friction coefficient; *L* be the coefficient; *c* be the diameter of the polished rod; *f* be the effective height of the sealing; *T*_*τ*_ be the tubing pressure; *T*_*s*_ be the power of the polished rod. Then, the transmission efficiency of the sealing device can be calculated by

(5) $$\begin{array}{c} \delta_{h}=100\frac{\left\{T_{s}-\left(3.1\times 10^{3}{\text{gLcfT}}_{\tau }u\right)\right\}}{T_{s}}. \end{array}$$

The power loss of the deep well pump mainly covers three parts: the power loss induced by mechanical friction, the leakage power loss of the pump, and the hydraulic power loss of the pump. Let *c*_1_ and *k* be the diameter and length of the plunger, respectively; Δ*t* be the difference between upper and lower pressures of the plunger; *ξ* be the radial gap between the plunger and the steel drum; *λ* be the viscosity of the well liquid; *σ* be the eccentric ratio; *ρ* be the eccentricity. Then, the power loss induced by mechanical friction of the deep well pump can be calculated by

(6) $$\begin{array}{c} \Delta T_{j}=\frac{\pi c_{1}mE}{6\times 10^{4}}\left[\frac{10^{60}\Delta t\xi }{2}+\frac{k\lambda mE}{60\xi \sqrt{1-\sigma^{2}}}\right]. \end{array}$$

The leakage power loss of the pump can be calculated by

(7) $$\begin{array}{c} \Delta T_{k}=\frac{10^{9}\pi c\Delta T^{2}\xi^{2}}{24\lambda k}\left(1+1.5\rho^{2}\right). \end{array}$$

Let *γ* be the drag coefficient of the well fluid passing through the flow valve bank; *φ* be the density of the well fluid; *W* be the flow of the well fluid passing through the pump valve orifice; and *χ* be the size of the orifice. Then, the hydraulic power loss of the pump can be calculated by

(8) $$\begin{array}{c} \Delta T_{q}=10^{-3}\gamma \phi \frac{W^{3}}{2\chi^{2}}. \end{array}$$

The power loss of the tubing includes leakage power loss and hydraulic power loss of the tubing. Let Δ*t* be the pressure difference between tubing and casing; *W* be the wellhead production of the oil well; and *W* be the displacement of the deep well pump. Then, the leakage power loss of the tubing can be calculated by

(9) $$\begin{array}{c} T_{hk}=10^{3}\Delta t\left(W-W_{y}\right). \end{array}$$

Let *i* be the grade number of sucker rod; *μ* be the friction factor of the tubing corresponding to grade *i* sucker rod; *K*_*i*_ be the length of grade *i* sucker rod; *c*_*ic*_ be the equivalent inner diameter of the tubing corresponding to grade *i* sucker rod; *v*_*i*_ be the well fluid speed corresponding to grade *i* sucker rod; and *W* be the flow of the tubing. Then, the hydraulic power loss of the tubing can be calculated by

(10) $$\begin{array}{c} \Delta T_{\tau }=10^{-3}\sum_{i=1}^{m}\mu_{i}\phi W\frac{K_{i}v_{i}}{2c_{ic}}. \end{array}$$

Let *W* be the daily fluid production of the pumper; *F* = *F*_*c*_ + 1000(*T*_*τ*_ − *T*_*r*_)/*φh* be the effective lift of the pumper; *F*_*c*_ be the depth of the dynamic liquid depth; *T*_*τ*_ and *T*_*r*_ be the pressures of the tubing and casing, respectively. Then, the effective power of the pumper can be expressed as follows:

(11) $$\begin{array}{c} T_{e}=\frac{WF\phi h}{86400}. \end{array}$$

Considering the components of beam pumper, the system efficiency was considered as the integration of the above aspects. If the efficiency is too low in any aspect, the overall efficiency of beam pumper will be influenced. In terms of motor factors, it is necessary to consider the specification, power, working voltage, and power factor of the motor. In terms of belt rotation, it is necessary to consider the following issues: the size of the belt, the matching between wheels and grooves, the suitability of the degree of tightness, and the cleanness of the belt. In terms of reduction box operation, it is necessary to consider the sufficiency and quality of gear oil, the intactness of components, and the smoothness of the oilway. In terms of sealing device, it is necessary to consider the alignment of the horsehead, the matching between sealing method and wellhead, and the degree of airtightness. In terms of the sucker rod, it is necessary to consider the timely cleaning of wax, punctual adjustment/replacement of the centering device, and the utilization of large tubing. In terms of deep well pump and tubing, it is necessary to consider implementing maintenance on a timely basis.

Through the above analysis on the balance and energy saving theory of the beam pumper, the following criteria were selected for evaluating practical application: changing the operating parameters of electrification, load torque, power frequency, load rate, and power factor; changing the transmission mode of the pumper to reduce the oscillation of the net torque; and adopting a structural balancing device for the pumper.

Figure 2 explains the flow of beam pumper model optimization. According to the calibration principle of steady-state system efficiency, the model optimization of beam pumper roughly contains four steps: model construction and scheme design, system efficiency calibration and correction, surface and downhole working condition calibration, and model optimization and verification. To improve the efficiency of the pumper, it is necessary to determine the order between efficiency correction and calibration according to the actual situation, or to perform them simultaneously.

## 3. RBF-Based Optimization

To enhance system efficiency by optimizing model parameters, this study obtains model samples through a reasonable design of beam pumper and train an RBF neural network based on these samples. Then, the authors set up the mapping relationship between the model parameters of beam pumper, which are identified in the preceding section, and the optimization objective (system efficiency). The purpose is to lower pumper energy consumption and improve the system efficiency of beam pumper.

The topology of RBF neural network is inspired by the perception ability of the retina.  Figure 3 shows the structure of RBF neural network. Let *a* be the input; *D*_*i*_ be the center of the receptive field of retinal neurons; *H*(.) be the radial basis activation function. Then, the signal outputted by retinal neurons can be characterized by the following function:

(12) $$\begin{array}{c} \Phi_{i}=H\left(\left\|a-D_{i}\right\|\right). \end{array}$$

The transfer function between input layer and hidden layer is usually defined as a Gaussian distribution function. Let *m* be the number of input layer nodes, *j* = 1, 2, 3,…, *m*, *l* = 1, 2, 3,…, *m*; *M* be the number of output layer nodes; *D*_*i*_ be the data at node *i* in the hidden layer; *ε*_*i*_ be the width of the first node in the hidden layer, *i* = 1, 2, 3,…, *t*; *t* be the number of hidden layer nodes; *a*_*l*_ − *D*_*i*_ be the Euclidean distance between *a*_*l*_ and *D*_*i*_; *θ*_*ij*_ be the weight from the *i*-th hidden layer node to the *j*-th output layer node. Then, the transfer function from the input layer to the output layer of RBF neural network can be expressed as follows:

(13) $$\begin{array}{c} b_{Lj}=\sum_{i=1}^{t}\theta_{ij}\exp^{\left(a_{l}-D_{i}/2\varepsilon_{i}\right)}. \end{array}$$

The above analysis shows that RBF neural network mainly consists of *D*_*i*_, *ε*_*i*_, and *θ*_*ij*_.

The hidden layer nodes of RBF neural network can be obtained through k-means clustering (KMC) through the following steps:

Step 1. Select *t* random cluster heads *D*_*i*_ from *w* samples of model parameters of beam pumper. For any sample *a*_*n*_, the class *λ*^(*n*)^ of the sample can be calculated by
  (14) $$\begin{array}{c} \lambda^{\left(n\right)}=\arg\underset{i}{\min}{\left\|a_{n}-D_{i}\right\|}^{2}. \end{array}$$
Step 2. Define the class of the cluster head, which is the closest to sample *a*_*n*_, out of the *t* cluster heads as *λ*^(*n*)^. Let *D*_*i*_ be that cluster head. Based on the calculation results of *λ*^(*n*)^, the head *D*_*i*_ of the class can be recalculated by
  (15) $$\begin{array}{c} D_{i}=\frac{\sum_{n=1}^{w}1\left\{\lambda^{\left(n\right)}=i\right\}a_{n}}{\sum_{n=1}^{w}1\left\{\lambda^{\left(n\right)}=i\right\}}. \end{array}$$

Repeat the above two steps until the cluster head changes very little, that is, the cluster head no longer changes, thereby determines the hidden layer nodes of the proposed network.

Let *ζ*_*i*_ be the minimum Euclidean distance between the *i*-th hidden layer node and other nodes; *υ* be the overlapping coefficient. Then, the node width *ε*_*i*_ can be determined by

(16) $$\begin{array}{c} \zeta_{i}=\min\left\|D_{i}-D_{g}\right\|,\\ \varepsilon_{i}=\upsilon \zeta_{i}. \end{array}$$

After *D*_*i*_ and *ε*_*i*_ are determined, the weight *θ*_*ij*_ can be obtained by the pseudo-inverse matrix method, according to the inputted model parameters and outputted optimized parameters of network training.

In actual practice, the hidden layer nodes of the RBF neural network obtained through KMC face several problems: the clustering results are significantly affected by the initial nodes, the clustering may fall into the local optimal trap, and the training algorithm could not converge. To avoid these problems and diversify hidden layer nodes, this study introduces the niche-sharing technique to determine the *t* hidden layer nodes *D*_*i*_ among the *w* model parameters.

In the niche-sharing mechanism, the Euclidean distance between individuals *a*_*i*_ and *a*_*j*_ is denoted as *ζ*_*ij*_; the niche radius is denoted as *ε*_*mic*_; the adjustment constant of the sharing function is denoted as *ϕ*. For individuals *a*_*i*_ and *a*_*j*_ in the population, the sharing function can be defined as follows:

(17) $$\begin{array}{c} \zeta_{ij}=\left\|a_{i}-a_{j}\right\|,\\ h\left(\zeta_{ij}\right)=\left\{\begin{array}{cc} 1-{\left(\frac{\zeta_{ij}}{\varepsilon_{\text{mic}}}\right)}^{\varphi }, & \zeta_{ij}<\varepsilon_{\text{mic}},\\ 0b, & \zeta_{ij}\geq \varepsilon_{\text{mic}}. \end{array}\right. \end{array}$$

For a niche containing *l* individuals, the sharing degree *e*_*i*_ of individual *a*_*i*_ in the population can be defined as follows:

(18) $$\begin{array}{c} e_{i}=\sum_{j=1}^{l}sh\left(\zeta_{ij}\right). \end{array}$$

Let *g*_*i*_ be the initial fitness of *a*_*i*_. Then, the sharing fitness *g*_  *i*_′ of that individual can be expressed as follows:

(19) $$\begin{array}{c} g_{i}^{\prime }=\frac{g_{i}}{e_{i}}. \end{array}$$

Based on the niche-sharing technique, the *t* hidden layer nodes *D*_*i*_ can be determined as follows:

To derive the sharing degree *SD*(*ζ*_*nm*_) between any two model parameter samples *a*_*n*_ and *a*_*m*_ of beam pumper, the first step is to compute the Euclidean distance *ζ*_*nm*_ between them:

(20) $$\begin{array}{c} \zeta_{nm}=\left\|a_{n}-a_{m}\right\|. \end{array}$$

The sum Ψ of the Euclidean distances between *a*_*n*_ and other samples can be calculated by

(21) $$\begin{array}{c} \Psi_{n}=\sum_{m=1}^{w}\left\|a_{n}-a_{m}\right\|. \end{array}$$

The niche radius *ε*_*mic*_ can be calculated by

(22) $$\begin{array}{c} \varepsilon_{mic}=\frac{\max\left(\phi_{n}\right)}{\sqrt{w}}. \end{array}$$

*SD*(*ζ*_*nm*_) can be calculated by

(23) $$\begin{array}{c} S\;D\left(\zeta_{nm}\right)=\left\{\begin{array}{cc} 1-\frac{\zeta_{nm}}{\varepsilon_{\text{mic}}}, & \zeta_{nm}<\varepsilon_{\text{mic}},\\ 0, & \zeta_{nm}\geq \varepsilon_{\text{mic}}. \end{array}\right. \end{array}$$

For any sample *a*_*n*_, the sharing degree *e*_*n*_ can be calculated by

(24) $$\begin{array}{c} e_{n}=\sum_{m=1}^{w}S\;D\left(\zeta_{nm}\right). \end{array}$$

The sharing fitness *g*_*i*_′ of sample *a*_*n*_ can be calculated by

(25) $$\begin{array}{c} g_{n}^{\prime }=\frac{\phi_{n}}{e_{n}}. \end{array}$$

Finally, *g*_*n*_′ values are ranked in descending order, and the *t* samples with the greatest *g*_*n*_′ are chosen as the hidden layer nodes *D*_*i*_ of the proposed neural network.

## 4. Experiments and Results Analysis

Table 1 summarizes the contents of model optimization for beam pumper.  Table 2 lists the prediction results on the model optimization parameters.

According to the schemes in Table 2, the improved beam pumper had smaller torques and cyclic load coefficient than the original machine. The mean input power of the motor can be obtained by the formulas in the preceding sections. The saved electrical energy is the energy consumption corresponding to the mean active power reduced by the falling cyclic load coefficient.

The following conclusions can be drawn from the analysis on the model optimization schemes of beam pumper: the power phase difference factor of the motor is inversely proportional to the periodic load coefficient, because the reduction of the factor lowers the difference. The various measures of model optimization all contribute to energy saving. The only difference lies in the hanging point load and the initial value. Model optimization schemes like adding a balancing device does not change the size of the rod, or the stroke of the pumper. But the other optimization measures can reduce the hanging point load, directly reducing the load of the pumper, and indirectly increasing the operation time and safety level of the machine.

Figures 4 and 5 present the torque curves of surface and downhole component optimization schemes, respectively. The three curves represent the mean torque, the maximum torque, and the minimum torque. According to the actual well condition specified by Yang et al. [25], the best choices are beam balancing, and adopting double horseheads.

It can be observed that the beam pumper after the model optimization through system efficiency analysis differed slightly in performance from the original beam pumper, but the optimized beam pumper achieved more stable torque curves, and ideal torque conditions.

This study prepares a training set of 500 parameter samples and a test set of 100 samples, which are related to beam pumper model. The small test set may lead to overfitting. To solve the problem, cross validation was carried out to optimize the model. Since system efficiency is the optimization objective, the error and precision of the output efficiency of our model were selected as the metrics of model prediction performance.  Figure 6 compares the actual system efficiency and predicted system efficiency in different groups of test samples. The system efficiency was predicted well at any sample.  Figure 7 compares the predicted errors of different test groups. Obviously, the mean absolute errors (MAEs) were mostly smaller than 1. A few test groups had a slightly large MAE because the system energy consumption varies with working conditions. But the overall errors are desirable.

After finalizing the model of our neural network, the outliers were removed from the verification points of system efficiency.  Figure 8 shows the errors between actual and predicted system efficiencies. It can be seen that the predicted system efficiencies on the test set were not very different from the actual values, and the output points were near the straight line of actual values. Hence, the proposed neural network boasts a good fitting effect, and a high prediction precision.

The experimental results show that the proposed optimization scheme basically achieved the expected effect, especially on consumption reduction and efficiency improvement. However, the stability, reliability, and energy-efficiency of the scheme in actual application need to be further tested. After the improved beam pumper operated stably for several hours, the current, power, and efficiency of the entire device were measured. The results show that the energy-efficiency of the improved device fell short of expectations, and only 11.5% of electricity was saved, compared to the original beam pumper. Besides, the rear balancing weight of the beam is quite heavy in the weight balancing structure. It adds to the difficulty for oil production engineers to complete the balancing operation, and slightly reduces security. Nevertheless, the proposed scheme is advantageous in terms of low retrofitting cost and high time efficiency.

## 5. Conclusion

This study puts forward an optimization approach for the model of beam pumper. First, the system efficiency of beam pumper was decomposed, the surface and downhole working efficiencies of beam pumper were analyzed, and the flow of beam pumper model optimization was clarified. Next, the model samples of beam pumper were adopted to train the proposed RBF neural network, and the mapping relationship was established between model parameters and the optimization objective (system efficiency). Through experiments, the authors summed up the contents of model optimization for beam pumper, predicted the model optimization parameters, and drew the torque curves of surface and downhole component optimization schemes, revealing that the optimized beam pumper achieved more stable torque curves, and ideal torque conditions. Finally, the system efficiencies were obtained at each test sample in different groups, the predicted errors of different test groups were compared, and the predicted system efficiencies were contrasted with the actual efficiencies. The results show that the proposed neural network boasts a good fitting effect, and a high prediction precision.

## Figures and Tables

**Figure 1:** Model structure of beam pumper.

**Figure 2:** Flow of beam pumper model optimization.

**Figure 3:** Structure of RBF neural network.

**Figure 4:** Torque curve of surface component optimization scheme.

**Figure 5:** Torque curve of downhole component optimization scheme.

**Figure 6:** System efficiencies in different groups of test samples.

**Figure 7:** A comparison of prediction errors of different test groups.

**Figure 8:** Errors between actual and predicted system efficiencies.

**Table 1:** Contents of model optimization.

Schemes	Main contents	Cycle	Cost
Surface component optimization scheme	Adjust motor specification; replace part of the belt, adjust wheel-groove matching degree, adjust belt tightness, and clean the belt; add gear oil to reduction box, clean oilway of reduction box, and check the intactness of box components; check the lubrication of rod mechanism	21 hours	70,000 yuan
Downhole component optimization scheme	Adjust tilt angle of horsehead, match sealing method with wellhead, and adjust sealing tightness; clean the wax, adjust/replace the centering device, and change for a large tubing; maintain deep well pump and tubing	166 hours	170,000 yuan

**Table 2:** Predicted optimization parameters.

Schemes	Polished rod load	Peak torque of reducer	Maximum negative torque	Root-mean-square matrix
Preoptimization	6.325 × 10^4^ N	4.015 × 10^4^ Nm	1.367 × 10^4^ Nm	1.846 × 10^4^ Nm
Scheme 1	6.271 × 10^4^ N	3.625 × 10^4^ Nm	1.146 × 10^4^ Nm	1.638 × 10^4^ Nm
Scheme 2	6.428 × 10^4^ N	2.738 × 10^4^ Nm	1.085 × 10^4^ Nm	1.148 × 10^4^ Nm
Scheme 3	5.649 × 10^4^ N	2.817 × 10^4^ Nm	0.64 × 10^4^ Nm	1.075 × 10^4^ Nm

Schemes	Cyclic load coefficient	Rated power of motor	Stroke	Stroke number
Preoptimization	1.625	13.25 kW	4 m	5
Scheme 1	1.473	12.47 kW	2 m	3
Scheme 2	1.395	8.47 kW	2 m	3
Scheme 3	1.42	7.49 *kW*	4 m	5

## Data Availability

The data used to support the findings of this study are available from the corresponding author upon request.

## References

[1] Qi X. Experiment researches of power equilibrium technology for beam pumping unit.

[2] Wang B. (2021). Dynamic strength analysis of the key components of the beam-type pumping unit with dynamic tracking balance. *Frattura Ed Integrità Strutturale*.

[3] Ging Y., Zhou H. P., Hu S. H. (2018). Application of beam pumping unit directly driven by permanent magnet integrated motor. *Acta Petrolei Sinica*.

[4] Wu J., Wang Q., Han Y. (2017). Finite element analysis of walking beam of a new compound adjustment balance pumping unit. *IOP Conference Series: Materials Science and Engineering*.

[5] Li K., Han Y. Diagnose for downhole working conditions of the beam pumping unit based on 16-directions chain codes and K-means clustering method.

[6] Zhao H. J., He K. K., Hu D. X., Lu M. (2021). Research on the soft-sensing method of polished rod load of beam pumping unit. *Chinese Journal of Scientific Instrument*.

[7] Feng Z.-M., Guo C., Zhang D. (2020). Variable speed drive optimization model and analysis of comprehensive performance of beam pumping unit. *Journal of Petroleum Science and Engineering*.

[8] Zhang C., Wang L., Li H. (2020). Optimization method based on process control of a new-type hydraulic-motor hybrid beam pumping unit. *Measurement*.

[9] Zhang C., Wang L., Zhao H., Wang L. Simulation research on hydraulic energy regulation system of beam pumping unit.

[10] Wang K., Gong G., Shen R. (2019). Novel physical network algorithm for indirect measurement of polished rod load of beam‐pumping unit. *Journal of Engineering*.

[11] Tan C., Feng Z.-M., Liu X. (2020). Review of variable speed drive technology in beam pumping units for energy-saving. *Energy Reports*.

[12] Liang Y., Wang T., Wang X., Liang W., Liu X. (2016). Simulation research on hydraulic hybrid assistant beam pumping unit. *Proceedings of the Institution of Mechanical Engineers - Part C: Journal of Mechanical Engineering Science*.

[13] Li K., Han Y., Wang T. (2018). A novel prediction method for down-hole working conditions of the beam pumping unit based on 8-directions chain codes and online sequential extreme learning machine. *Journal of Petroleum Science and Engineering*.

[14] Huang J. L., Wang Y. F., Dang X. W. (2013). Kinematics analysis and simulation of main components of beam pumping unit based on matlab. *Advanced Materials Research*.

[15] Feng Z. M., Li Q., Xu Y., Liu B. W. (2013). Kinematics analysis of beam pumping unit base on projection method. *Journal of Chemical and Pharmaceutical Research*.

[16] Feng Z.-M., Tan J.-j., Liu X., Fang X. (2017). Selection method modelling and matching rule for rated power of prime motor used by beam pumping units. *Journal of Petroleum Science and Engineering*.

[17] Li K., Han Y., Li S. M., Wang T. (2017). OS-ELM-based hybrid online modeling for motor load torque of beam pumping units. *CIESC Journal*.

[18] Lu J., He J., Mao C., Wu W., Wang D., Lee W.-J. (2014). Design and implementation of a dual PWM frequency converter used in beam pumping unit for energy saving. *IEEE Transactions on Industry Applications*.

[19] Li X. G., Xiao P. P. (2014). Study of energy saving controller for beam pumping unit base on Neural Net PID. *Applied Mechanics and Materials*.

[20] Xing M. M., Dong S. M. (2014). The simulation model of belt longitudinal vibration characteristics in beam pumping unit. *Journal of Vibration Engineering*.

[21] Li K., Han Y. (2018). Modelling for motor load torque with dynamic load changes of beam pumping units based on a serial hybrid model. *Transactions of the Institute of Measurement and Control*.

[22] Zi-Ming F., Jing-Jing T., Yanan S., De-Shi Z., Wei-Bo D. (2018). 3D-Dynamic modelling and performance analysis of service behavior for beam pumping unit. *Mathematical Problems in Engineering*.

[23] Gu X.-h., Liao Z.-q., Hu S., Yi J., Li T.-f. Decision parameter optimization of beam pumping unit based on BP networks model. *Fuzzy Information & Engineering and Operations Research & Management*.

[24] Li Y. B., Jiang T., Gao Y. H., Yu L. Y. (2012). Design optimization of beam-pumping unit based on improved particle swarm optimization. *Applied Mechanics and Materials*.

[25] Yang X. J., Yan T., Yan X. Z. (2011). Optimization design of beam pumping unit based on response surface method. *Advanced Materials Research*.

[26] Niu W. J. (2011). The research on modular and parametric design system for beam pumping unit. *Applied Mechanics and Materials*.

